RETRACTED

# Traumatic hemorrhage of occult phaeochromocytoma in a patient with septic shock

**DOI:** 10.4103/0974-2700.66549

**Published:** 2010

**Authors:** Mohammad Shahnawaz Moazzam, Syed Moied Ahmed, Shahjahan Bano

**Affiliations:** Department of Anaesthesiology & Critical Care, Faculty of Medicine, J.N. Medical College, AMU, Aligarh, U.P.-202 002, India

**Keywords:** Phaeochromocytoma, sepsis, traumatic haemorrhage

## Abstract

Phaeochromocytoma can have a variety of presentations; however, traumatic hemorrhage into a phaeochromocytoma is a very rare presentation. Diagnosing and managing a critically ill, septic patient with a Phaeochromocytoma can be very challenging. We report a case of 53 years old man with a previously undiagnosed Phaeochromocytoma, who presented initially with bowel perforation following an assault. Following a laparotomy for bowel resection and anastomosis, whilst on the intensive care unit, he developed paroxysmal severe hypertension overlying septic shock. Phaeochromocytoma was confirmed using a computed tomography scan and urinary assay of metanephrine and catecholamines. We managed the haemodynamic instability using labetalol and noradrenaline infusions. As his septic state improved he was convention therapy and following control of his symptoms over the next few weeks, he underwent an uncomplicated right sided adrenalectomy. He made a full recovery.

## INTRODUCTION

Phaeochromocytoma is a rare tumour of the chromaffin cells arising most commonly from the adrenal medulla. They typically present with hypertension and a characteristic symptom triad of headache, diaphoresis and palpitations. They are however known to be a great mimic and may have a variety of other presentations. Latent phaeochromocytomas has presented as hypertensive crises during anaesthesia and surgery,[1] acute abdomens,[2] multiple organ failure,[3] cardiac failure, myocardial infarction and stroke.[4] Cases of traumatic haemorrhage of a phaeochromocytoma resulting in its presentation,[5] have also been previously described.

We report a case of an undiagnosed phaeochromocytoma which presented as a hypertensive emergency 5 days after an assault. The patient had already safely undergone an emergency laparotomy during this period, but the tumour had not manifest until he became septic during the postoperative period. We discuss the clinical dilemma of managing a critical ill, septic patient with paroxysmal hypertension because of a stimulated phaeochromocytoma.

## CASE HISTORY

A case of a 53 year old man presented to our emergency department with abdominal pain following an assault 16 hours previously. His medical history was unremarkable except for moderate alcohol intake and his surgical history included an uneventful laparoscopic cholecystectomy. A diagnosis of peritonitis followed by bowel perforation was made and he underwent an emergency laparotomy under general anaesthesia. He remained cardiovascularly stable throughout the procedure. The systolic arterial pressure (SAP) range between 90 and 140 mmHg and his heart rate ranged between 90 and 110 per minute. A short segment of perforated ileum was resected and an end-to-end anastomosis performed. Patient was reversed from general anaesthesia and shifted to postoperative ward. After two days, he appeared increasingly unwell with sputum retention and suspected sepsis. He was shifted to intensive care unit (ICU) from surgical ward and a decision was made to re-intubate. Induction of anaesthesia was performed with propofol and rocuronium. Sedation was maintained using midazolam infusions. Following tracheal intubation his arterial pressure increased to 326/142 mmHg. The cardiovascular response was initially presumed to be an exaggerated pressure response to intubation, and further boluses of propofol were administered. Despite adding high dose of propofol his SAP remained in the range of 240-340 mmHg. At this point a glyceryl trinitrate (GTN) infusion was added to manage the hypertensive crises. For the next few hours the mean arterial pressure (MAP) swung between 224 and 44 mm Hg. This raised the possibility of a phaeochromocytoma and septic shock. A labetalol infusion was started and GTN was reduced. The hypotensive episodes required the administration of noradrenaline. A contrast-enhance computed tomography (CECT) scan of the abdomen demonstrated a 5.5 cm lesion originated from the right adrenal gland suggesting the possibility of haemorrhage within an adrenal tumour [Figure 1]. Serum and urinary biochemical test were sent before the exogenous administration of noradrenaline. He remained septic, raising the possibility of an anastomotic breakdown, necessitating a return to the operation theatre. Anaesthetic plans for cardiovascular instability were made but his haemodynamic parameters remained stable throughout the procedure. Anastomotic breakdown was confirmed and end ileostomy was performed. With resolution of his intra-abdominal sepsis his gut function improved and enteral phenoxybenzamine was commenced and labetalol was reduced. He recovered enough to be discharged back to the surgical ward after a 22-day stay in ICU. The phenoxybenzamine dose was slowly increased to 80 mg twice a day and atenolol was also added. Five weeks later the ileostomy closure was done and a right adrenalectomy was performed. He remained cardiovascularly stable throughout the perioperative period. The histopathology of the gland confirmed the presence of haemorrhagic necrosis into a phaeochromocytoma [Figure 2a, 2b].

RETRACTED

**Figure 1:** CECT-scan of abdomen showing tumour arising from the right adrenal gland with streaking of fat posterior to the tumour suggesting haemorrhage (arrow)

**Figure 2:** Histopatological slides of the excised adrenal mass showing, (a) tumour gland showing large areas of necrosis: (b) tumour showing features of phaeochromocytoma. Note the “Zellballen pattern” composed of rounded nests of cells separated by thin-walled blood vessels and scattered atypical giant cells

## DISCUSSION

Phaeochromocytomas are responsible for hypertension in about 0.1% of those presenting with hypertension. Although they typically arise from the adrenal medulla, they may develop from chromaffin cells in or around sympathetic ganglia as well. Ninety percent are unilateral, predominantly right sided. Ten percent of familial cases follow an autosomal dominant pattern of inheritance and occur either alone or in combination with multiple endocrine neoplasia (MEN)-2a, MEN-2b, Von Reck-linghausen’s disease or Von Hipple Lindau retinal cerebellar haemangioblastoma. About 10% of phaeochromocytomas in adult are extra-adrenal and are more likely to be malignant. The other common symptoms include headache, sweating, palpitation, nervousness, nausea and vomiting, abdominal pain and weakness.[6] On questioning this patient following his recovery, he had no such complaints before this hypertensive episode.

Traumatic adrenal haemorrhage, resulting in the manifestations of a phaeochromocytoma, is a very rare. Traumatic adrenal haemorrhage, without a phaeochromocytoma may itself present as a hyper-adrenergic state, but then tends to improve as the haematoma resolves and the gland resumes normal function. Complete destruction of adrenals following injury or haemorrhage is likely to produce adreno-cortical insufficiency resulting in shock.[7]

Faced with severe hypertension, we initially treated the more probable causes in such a situation. The possibility of inadequate sedation or analgesia was managed by increasing the dose of sedation and analgesic agents. In a previously normotensive patient with no underlying renal dysfunction, and improbable drug interaction, the possibility of an underlying endocrine disorder was more likely. The magnitude of the raised blood pressure and the difficulty in controlling it with propofol and GTN; suggested an intense catecholamine response, i.e., a phaeochromocytoma. An α-blocking agent is the drug of choice for hypertensive crisis in these situations with or without a β-blocker added to combat reflex or associated tachycardia. We chose to use labetalol because of it’s combined α- and β-receptor blocking abilities, and also due to the fact that enteral administration of phenoxybenzamine was not possible because of bowel trauma. Labetalol worked well in controlling the hypertensive episodes but the underlying septic shock required a noradrenaline infusion. Our patient had both a noradrenaline and adrenaline secreting tumour with hypertension and tachycardia as well, so we considered combined α- and β-receptor blockade. Subsequently, our patient was started on conventional; oral phenoxybenzamine:- a long acting, non-selective α-receptor blocking drug, with a later addition of atenolol.

RETRACTED

The presence of hypotension, requiring noradrenaline infusion raised the possibility of a septic shock. The evidence in favour of sepsis-induced shock included a raised total leukocytes counts (TLC) and acute phase reactants on the background of a recent intra-abdominal pathology requiring surgery. Predominantly adrenaline secreting tumours may present with a “septic shock” kind of picture. However, in our case, the urinary analysis revealed grossly elevated noradrenalin and adrenaline levels suggesting a tumour secreting both the catecholamines. Phaechromocytomas may also cause a hypertensive cardiomyopathy resulting in cardiac failure,[8] but in our case evidence of a hyperdynamic circulation (↑ cardiac index and ↓ systemic vascular resistance) requiring vasopressures rather than inotropes supported the diagnosis of septic shock. The diagnosis of phaeochromocytoma was made following a CECT scan study and assay of the urinary catecholamines and their metabolites. Twenty-four hours urinary catecholamine levels; and total metanephrine level; have consistently proven to be the most specific tests available for the diagnosis of phaeochromocytoma (sensitivity 89% and specificity 99%).[9] The diagnosis in our patient was confirmed by the presence of haemorrhage necrosis of a phaeochromocytoma in the histology of gland.

## CONCLUSIONS

Phaeochromocytoma discovered during the management of an unrelated illness is a rare presentation of these tumors. We have reported an unusual case of traumatic hemorrhage of occult pheochromocytoma, presenting with severe labile hypertension and associated with septic shock. Diagnosing and managing a critically ill, septic patient with a Phaeochromocytoma can have very challenging. Because the key to diagnosing and managing the phaeochromocytoma in a septic shock patient,: 1) presence of severe and labile hypertension could not control with the administration of propofol and GTN postoperative period and managed with administration of labetalol; 2) raised TLC and Acute phase reactant with episode of hypotension managed with infusion of noradrenaline. Remarkably, above clinical scenarios were present in our patient in addition to the rare and serious complication of traumatic hemorrhage of adrenal tumour with sepsis.

RETRACTED

## References

[1] Dabbous A, Siddik-Sayyid S, Baraka A (2007). Catastrophic hemodynamic changes in a patient with undiagnosed pheochromocytoma undergoing abdominal hysterectomy. Anesth Analg.

[2] Hatada T, Nakai T, Aoki I, Gondo N, Katou N, Yoshinaga K (1994). Acute abdominal symptoms caused by hemorrhagic necrosis of pheochromocytoma: report of a case. Surg Today.

[3] Kolhe N, Stoves J, Richardson D, Davison AM, Gilbey S (2001). Hypertension due to phaeochromocytoma- an unusual cause of multiorgan failure. Nephrol Dial Transplant.

[4] Kanjaa N, Khatouf M, Elhijri A, Harrandou M, Azzouzi A, Benerradi H (1999). Pheochromocytoma, Sever and uncommon presentations. Ann Fr Anesth Reanim.

[5] May EE, Beal AL, Beilman GJ (2000). Traumatic hemorrhage of occult pheochromocytoma: a case report and review of the literature. Am Surg.

[6] Jalbout M, Siddik-Sayyid S, Baraka A (2003). Perianesthetic management of patients undergoing resection of pheochromocytoma. Middle East J Anesthesiol.

[7] Guichelaar MM, Leenen LP, Braams R (2004). Transient adreno-cortical insufficiency following traumatic bilateral adrenal hemorrhage. J Trauma.

[8] Kassim TA, Clarke DD, Mai VQ, Clyde PW, Mohamed Shakir KM (2008). Catecholamine-induced cardiomyopathy. Endocr Pract.

[9] Harding JL, Yeh MW, Robinson BG, Delbridge LW, Sidhu SB (2005). Potential pitfalls in the diagnosis of phaeochromocytoma. Med J Aust.

